# Cinnamic Acid Ameliorates Nonalcoholic Fatty Liver Disease by Suppressing Hepatic Lipogenesis and Promoting Fatty Acid Oxidation

**DOI:** 10.1155/2021/9561613

**Published:** 2021-09-02

**Authors:** You Wu, Minghui Wang, Tao Yang, Lingling Qin, Yaomu Hu, Dan Zhao, Lili Wu, Tonghua Liu

**Affiliations:** ^1^Key Laboratory of Health Cultivation of the Ministry of Education, Beijing University of Chinese Medicine, Beijing 100029, China; ^2^Key Laboratory of Health Cultivation of Beijing, Beijing University of Chinese Medicine, Beijing 100029, China; ^3^Chengdu Integrated TCM and Western Medicine Hospital, Chengdu 610016, China; ^4^Department of Science and Technology, Beijing University of Chinese Medicine, Beijing 100029, China; ^5^First School of Clinical Medicine, Shaanxi University of Chinese Medicine, Xianyang 712046, China

## Abstract

**Background:**

Cinnamic acid (CA) has been shown to have many beneficial effects including regulating lipid metabolism and reducing obesity. However, its effect on nonalcoholic fatty liver disease (NAFDL) has not been investigated in detail. Thus, we performed this study in order to explore CA's effect on hepatic lipid metabolism and the underlying mechanisms.

**Method:**

Oleic acid (OA) was used to induce lipid accumulation in HepG2 cells. After coincubation with CA, the cells were stained with oil red O and the triglyceride (TG) content was assessed. Key genes in lipogenesis and fatty acid oxidation pathways were tested. Additionally, db/db and wt/wt mice were divided into three groups, with the wt/wt mice representing the normal group and the db/db mice being divided into the NAFLD and CA groups. After 4 weeks of oral treatment, all mice were sacrificed and the blood lipid profile and liver tissues were assessed.

**Results:**

CA treatment reduced the lipid accumulation in HepG2 cells and in db/db mouse livers. ACLY, ACC, FAS, SCD1, PPAR*γ*, and CD36 were significantly downregulated, while CPT1A, PGC1*α*, and PPAR*α* were significantly upregulated.

**Conclusion:**

CA's therapeutic effect on NAFLD may be attributed to its ability to lower hepatic lipid accumulation, which is mediated by suppression of hepatic lipogenesis and fatty acid intake, as well as increased fatty acid oxidation.

## 1. Introduction

Nonalcoholic fatty liver disease (NAFLD), the incidence of which often parallels the trends in obesity, type II diabetes, dyslipidemia, and other metabolic diseases, has become a major health problem worldwide and the most common chronic liver disease in recent years [1]. The global prevalence of NAFLD is approximately 25.24% [2] and the rate continues to increase [3]. NAFLD begins with simple hepatic steatosis and can develop into nonalcoholic steatohepatitis, potentially leading to hepatic fibrosis and cirrhosis and causing severe complications such as hepatocellular carcinoma [1]. It reflects disrupted body energy homeostasis, which is the common pathological change in metabolic diseases.

Intrahepatic triglyceride (IHTG) accumulation indicates imbalanced hepatic energy metabolism and it can be regarded as a biomarker of NAFLD [4, 5]. Abnormally high IHTG levels in individuals with NAFLD may be attributed to increased *de novo* lipogenesis (DNL) and decreased fatty acid oxidation. Fatty acids are synthesized in the liver through DNL and are esterified by glycerol-3-phosphate to produce triglyceride (TG). DNL is mediated by several lipogenic enzymes, the transcription of which is governed by transcription factors such as carbohydrate-responsive element-binding protein (ChREBP), sterol regulatory element-binding protein 1c (SREBP1c), and liver X receptors (LXRs) [6]. Fatty acid catabolism in the liver mainly takes place within mitochondria, generating ATP and ketone bodies. Long-chain fatty acid- (LCFA-) CoA translocates into mitochondria, which is mediated by carnitine palmitoyltransferase-1A (CPT1A), the rate-limiting enzyme for fatty acid *β*-oxidation [7]. Altered activity of the above pathways in individuals who consume excess calories results in NAFLD and other metabolic diseases [8]. Thus, regulating energy metabolism, especially the fatty acid synthesis and oxidation pathways in hepatocytes, plays an important role in controlling excess IHTG levels and, eventually, improves the condition of NAFLD.

Cinnamic acid (CA) is a natural polyphenol that comprises nine carbon atoms (C6-C3) (Figure 1(a)). It occurs in many fruits such as citrus fruits and grape and vegetables such as spinach and celery, and CA and its many derivatives are permitted to be used as flavor compounds in numerous regions by authorities [9, 10]. However, it is mostly enriched in *Cinnamomum cassia* (Chinese cinnamon) [11, 12], which has been used as a traditional herb as well as a flavoring material in many countries for thousands of years [13]. It has been demonstrated that CA possesses multiple therapeutic effects, including antimicrobial [14], anticancer [15, 16], anti-inflammatory [17], antioxidant [18, 19], and antidiabetic [10] effects. Moreover, recent studies have highlighted CA's effects on lipid metabolism and obesity. It was reported that CA lowered the serum lipid levels in streptozotocin- (STZ-) induced diabetic rats [20] and in animal models of high fat diet-induced obesity [21, 22]. *In vitro* studies showed that CA stimulated white fat browning in 3T3-L1 adipocytes and activated HIB1B brown adipocytes [23]. It also lowered the TG levels in 3T3-L1 cells [24] and lipid accumulation in oleic acid- (OA-) treated HepG2 hepatocytes [22]. Moreover, in a previous study on a palmitic acid-induced triglyceride accumulation cell model, CA treatment elevated CPT1 protein expression, suggesting CA may accelerate lipid oxidation *in vitro* [25].

Although CA has exhibited hypolipidemic effects in both *in vivo* and *in vitro* experiments, the underlying mechanisms of CA's effect on NAFLD are still poorly understood. Thus, we investigated the effect of CA on OA-stimulated HepG2 cells and db/db mice, a commonly used genetic model for NAFLD [26, 27], and we explored the alterations in the expression of transcription factors and key enzymes in the lipogenesis and fatty acid oxidation pathways in cells and mice after CA treatment.

## 2. Materials and Methods

### 2.1. Chemicals and Reagents

Cinnamic acid (≥99.5% purity) was purchased from Shanghai Yuanye (Shanghai, China). Dulbecco's modified eagle medium (DMEM), fetal bovine serum (FBS), and 0.25% trypsin-ethylenediaminetetraacetic acid (EDTA) were purchased from Gibco (Carlsbad, CA, USA). OA was purchased from Sigma-Aldrich (St. Louis, MO, USA). Bovine serum albumin (BSA) and 0.5% carboxymethyl cellulose (CMC) sodium salt solution were purchased from Solarbio Science & Technology (Beijing, China) and Coolaber Science & Technology (Beijing, China), respectively. CA was dissolved in 0.5% CMC buffer solution before being orally administered to the mice.

### 2.2. Cell Culture

HepG2 cells were purchased from KeyGEN Biotech (Nanjing, China). The cells were cultured in DMEM with 10% FBS and maintained in a humidified, 37°C, 5% CO_2_ environment, with the media changed every 24 hours. Based on previous studies, 0.5 mM OA was used to establish a high-fat model *in vitro* [28, 29]. After reaching 80% confluence, the cells were placed in 6-well plates and stimulated with 0.5 mM OA media with or without CA of different concentrations. Cells cultured without OA were used as normal controls. The OA/BSA complex used for cell stimulation was prepared as follows: OA was dissolved in 0.1 M NaOH and heated at 70°C for 30 min to form a 100 mM OA solution. This was further mixed with 10% BSA in phosphate-buffered saline to acquire a 10 mM OA/BSA complex. This complex was diluted in DMEM with 10% FBS to a concentration of 0.5 mM for final use. All cell experiments were performed in at least three replicate wells.

### 2.3. Cell Viability Assay

The effect of CA on the viability of HepG2 cells was assessed by Cell Counting Kit- (CCK-) 8 assays. CCK-8 assays were conducted as previously described [22, 30] with slight modification. Briefly, 200 *μ*l HepG2 cells were seeded at a density of 1 × 10^4^/well in a 96-well plate and cultured for 12 h. Thereafter, the cells were treated with CA (diluted to 12.5, 25, 50, 100, or 200 *μ*M) for 24 h, followed by changing the media to 200 *μ*L DMEM containing 10 *μ*L CCK-8 solution (Dojindo Molecular Technologies, Kumamoto, Japan) and incubating for 1 h in 37°C. Absorbance at 450 nm was measured using a microplate reader (Promega BioSystems Sunnyvale, Sunnyvale, CA, USA). Cells cultured in DMEM with 10% FBS (without CA) were used as normal controls.

### 2.4. Oil Red O Staining and TG Assessment

After treatment for 24 h, HepG2 cells were stained with Oil red O to determine the intracellular lipid accumulation. The staining was performed using a commercial kit (Solarbio Science & Technology) according to the manufacturer's instructions. TG content of HepG2 cells was determined using a TG measuring kit (Nanjing Jiancheng Bioengineering, Nanjing, China) following the manufacturer's instructions. Cells cultured in DMEM with 10% FBS were used as normal controls.

### 2.5. Animal Experiments

The animal experiments conducted in this study were approved by the Animal Care and Ethics Committee of Beijing University of Traditional Chinese Medicine (approval no. BUCM-4-20190931002-1088). A total number of 14 5-week-old male C57BL/KsJ-db/db mice and 7 age-matched male C57 BL/KsJ-wt/wt mice were purchased from Nanjing Biomedical Research Institute of Nanjing University (Nanjing, China) and housed in specific-pathogen-free conditions under a 12/12 h light/dark cycle, with free access to water and food. The bodyweight of mice was measured every week. After 1 week of acclimatization, all mice were fasted overnight and blood glucose was measured by a portable glucometer (Glucocard 01-mini; Arkray, Kyoto, Japan) using blood collected from the tail vein.

The db/db mice were then randomly divided into two groups with fasting blood glucose and body weight of which at the same baseline: the CA and NAFLD groups. The CA mice were orally treated with 20 mg/kg body weight CA every day. The dosage was chosen based on previous studies. The NAFLD model mice were treated with the same volume of the vehicle (0.5% CMC buffer). The wt/wt mice were used as the normal control group and treated the same as NAFLD mice. After 4 weeks of treatment, the mice were sacrificed. Blood samples were collected and centrifuged to acquire serum. Additionally, liver and epididymal adipose tissues were removed and weighed. A small slice of each tissue was fixed in 4% paraformaldehyde solution (Solarbio Science & Technology) and the remaining tissues were immediately frozen in liquid nitrogen.

### 2.6. Assessment of Serum Lipid Profile and IHTG

The serum was stored at −20°C before the total cholesterol (TC), TG, high-density lipoprotein (HDL), low-density lipoprotein (LDL), free fatty acid (FFA), and glucose levels were tested using an automated chemistry analyzer (AU480; Beckman Coulter, Brea, CA, USA). IHTG levels (mmol/g protein) of the mice were measured using a commercial kit (Nanjing Jiancheng Bioengineering, Nanjing, China).

### 2.7. Histological Analysis of Liver and Adipose Tissues

Liver tissues and epididymal adipose tissues fixed in 4% paraformaldehyde were embedded in paraffin, cut into 4 *μ*m thick slices using a microtome, and then stained with hematoxylin and eosin (H&E). Immunohistochemical (IHC) staining of liver tissues was used to examine protein expression. Primary antibodies against SREBP1 (ab191857; Abcam, Cambridge, UK) and CPT1A (ab234111; Abcam) were used, followed by incubation with horseradish peroxidase- (HRP-) labeled anti-rabbit IgG secondary antibody for 20 min. The tissues were then stained with 3,3′-diaminobenzidine (DAB) and counterstained with hematoxylin. The IHC staining images were analyzed based on the mean optical density using ImageJ software (National Institutes of Health, Bethesda, MD, USA).

### 2.8. Quantitative Real-Time PCR (RT-qPCR)

Total RNA was extracted from HepG2 cells and the liver tissues using a commercial kit (Tiangen Biotech, Beijing, China) according to the manufacturer's instructions. The RNA was then homogenized by RNase-free water to the same concentration of 0.5 ng/tube and cDNA was synthesized using a PrimeScript™ RT Reagent Kit with gDNA Eraser (Takara Bio, Kusatsu, Japan). Thereafter, the RT-qPCR analyses were conducted on Applied Biosystems 7500 Real-Time PCR system (Thermo Fisher Scientific, Waltham, MA, USA) using a GoTaq®qPCR Master Mix Kit (Promega). The expression levels of target genes were normalized to glyceraldehyde 3-phosphate dehydrogenase (GAPDH) and the results were calculated using the relative quantitative (2^−ΔΔCT^) method. The primers used are listed in Table 1.

### 2.9. Western Blot Analysis

Total protein was extracted from the liver tissues as follows. The tissues were homogenized and lysed using radioimmunoprecipitation assay (RIPA) lysis buffer containing protease inhibitor, phosphatase inhibitor, and phenylmethanesulfonyl fluoride (KeyGEN Biotech). The concentration of each extracted protein solution was then measured using a Bradford protein quantitative assay with Coomassie brilliant blue G-250 (Solarbio Science & Technology). Protein samples were prepared at a concentration of 1 *μ*g/*μ*l and denatured at 100°C for 5 min in loading buffer (Solarbio Science & Technology). The proteins were loaded onto 10% sodium dodecyl sulfate-polyacrylamide gel electrophoresis (SDS-PAGE) gels and separated according to their molecular weights. They were then transferred onto methanol-soaked 0.45 *μ*m polyvinylidene fluoride membranes (Millipore, Bedford, MA, USA). These membranes were then blocked using Blocking-One solution (Nacalai Tesque, Kyoto, Japan) for 1 h and then incubated with primary antibodies against the following proteins: ATP-citrate lyase (ACLY; #13390; Cell Signaling Technology, USA), acetyl-CoA carboxylase (ACC; #3676; Cell Signaling Technology), fatty acid synthase (FAS; #3180; Cell Signaling Technology), stearoyl-CoA desaturase 1 (SCD1; #2794; Cell Signaling Technology), CPT1A (ab234111; Abcam), and *β*-actin (#4970; Cell Signaling Technology) at 4°C overnight. After washing with Tris-buffered saline with Tween 20 (TBST; Beijing Applygen Technologies, Beijing, China), the membranes were incubated with HRP-conjugated AffiniPure goat anti-rabbit IgG secondary antibody (Proteintech Group, Rosemont, IL, USA) for 1 h and washed with TBST again. Enhanced chemiluminescence (ECL) reagent (Solarbio Science & Technology) was reacted with the HRP to generate fluorescence. The gray values of the protein bands were calculated by normalization to the endogenous control protein *β*-actin.

### 2.10. Statistical Analysis

All data are presented as mean ± standard deviation (SD). SPSS 23.0 software (SPSS, Chicago, IL, USA) was used for statistical analysis. Normally distributed data were compared between two groups using Student's *t*-test. Normally distributed data were compared between three or more groups using one-way analysis of variance (ANOVA) followed by the least significant difference (LSD) test for groups with equal variances or Dunnett's test for groups with unequal variances. Nonnormally distributed data were compared between two groups using the Mann-Whitney *U* test. Nonnormally distributed data were compared between three or more groups using the nonparametric Kruskal–Wallis test. A statistically significant difference was defined as *p* < 0.05 or *p* < 0.01.

## 3. Results

### 3.1. Effect of CA on HepG2 Cell Viability

CA treatment at doses of 12.5, 25, 50, or 100 *μ*M for 24 h had no significant impact on the viability of HepG2 cells (Figure 1(b)). The viability of the cells in the 200 µM CA group was lower than that of the control group (*p* < 0.05). Therefore, 25, 50, and 100 *μ*M CA were chosen for further investigations.

### 3.2. Effect of CA on Lipid Accumulation in HepG2 Cells

Oil red O staining showed that OA dramatically increased the lipid accumulation in HepG2 cells and CA treatment ameliorated this increase. The lipid droplets were remarkably reduced in the CA group compared to the NAFLD group (Figure 1(c)). This was further confirmed by the results of the TG content examination. The TG content was significantly increased by OA, and CA reduced the TG content in a dose-dependent manner (Figure 1(d)). qPCR results indicated that CA treatment significantly suppressed the expression of ACLY and FAS. It also showed the tendency to decrease the expression of ACC1, ACC2, and SCD1 and increase the expression of CPT1A (statistically insignificant, Figure 1(e)).

### 3.3. Effect of CA on Body Weight, Blood Glucose, and Liver and Fat Mass of db/db Mice

Mice in the CA group were lighter after 4 weeks than those in the NAFLD group (Figures 2(a) and 2(b)). Oral administration of CA significantly reduced body weight gain of db/db mice from the third week. Notably, CA decreased the liver mass and liver index (liver mass/body weight) in the obese db/db mice (*p* < 0.05 and *p* < 0.01, respectively) (Figures 2(c) and 2(d)). CA also exhibited a hypoglycemic effect in the db/db mice, as at the end of the treatment, the glucose levels in CA group were significantly lower than those in the NAFLD group despite the same baseline (Figure 2(e)), confirming its previously reported antidiabetic effect [31, 32]. Furthermore, CA reduced the mean weight of epididymal fat, though the data was not significant according to one-way ANOVA (Figure 2(f)).

### 3.4. Effect of CA on Serum Lipid Profile and IHTG Levels in db/db Mice

The serum TG, IHTG, and FFA levels in db/db mice were significantly lowered and the HDL level was raised by CA treatment (Figures 3(b), 3(c), 3(e), and 3(f)), suggesting that CA improved lipid metabolism and may have a beneficial effect on NAFLD. However, CA had no noticeable effect on serum TC or LDL levels (Figures 3(a) and 3(d)).

### 3.5. Histological Observation Results

The liver tissues and epididymal adipose tissues were fixed in paraffin and stained with H&E for observation of histological changes. Compared to normal wt/wt mice, db/db mice in the NAFLD group had severe hepatic steatosis and disruption of hepatocyte structure (Figure 4(a)). These changes were ameliorated by CA treatment. Adipocytes in the NAFLD group were dramatically larger than those in the normal control group, consistent with the abovementioned increased epididymal fat mass. H&E staining showed that 4 weeks of CA treatment reduced the size of the adipocytes (Figure 4(b)). The IHC analysis showed less SREBP1c-positive staining in the CA group than the NAFLD group (Figure 4(c)). In contrast, the CPT1A-positive area was larger in the CA group than the NAFLD group (Figure 4(d)). The IHC results were further quantified and verified based on mean optical density using ImageJ software (Figure 4(e)).

### 3.6. CA Downregulated Lipogenesis Transcription Factors and Lipogenic Enzymes in db/db Mice

The relative mRNA expression of transcription factors that regulate genes that encode lipogenic enzymes was downregulated and, consistently, the mRNA and protein expression of lipogenic enzymes including ACLY, ACC, FAS, and SCD1 were decreased (Figure 5). The mRNA expression of factors related to the expression and regulation of transcription factors, such as branched-chain ketoacid dehydrogenase kinase (BDK) and branched-chain ketoacid dehydrogenase phosphatase (PPM1K), was also investigated by qPCR. Moreover, BDK and PPM1K mRNA expression was decreased and increased by CA, respectively. This led to a significantly decreased BDK : PPM1K in the CA group.

### 3.7. CA Upregulated Fatty Acid Oxidation Pathway in db/db Mice

Compared to the NAFLD group, mice in the CA group had higher CPT1A protein expression, which indicates that fatty acid oxidation was upregulated in the CA group. Additional factors from fatty acid metabolism pathways were also examined by qPCR. The results showed that CA increased the mRNA expression of peroxisome proliferator-activated receptor *α* (PPAR*α*) and peroxisome proliferator-activated receptor-*γ* coactivator 1*α* (PGC1*α*) and decreased the mRNA expression of ACC2 and CD36 (Figure 6).

## 4. Discussion

As the most common chronic liver disease, NAFLD affects nearly one-third of the adult population and 10% of children in developed countries, and the prevalence continues to increase in concert with the increasing number of obese individuals [33, 34]. In Asian countries, the current prevalence of NAFLD is around 25%, which is also increasing [35]. Unhealthy lifestyles, especially overconsumption of high-calorie foods and sedentary lifestyles and lack of exercise, lead to disorders of energy metabolism, causing dyslipidemia, obesity, metabolic syndrome, and type 2 diabetes [36].

CA, a chemical almost ubiquitous in plants and particularly enriched in cinnamon, has been reported to improve lipid metabolism and ameliorate diabetes and obesity [20, 21, 23, 31, 32, 37–39]. Despite recent research progress, CA's effects on NAFLD and the possible mechanisms remain to be elucidated. The development of NAFLD is linked to the abnormal accumulation of hepatic lipids, manifested as an excessive level of IHTG [33]. In our study, CA treatment significantly decreased OA-induced lipid accumulation in HepG2 cells and significantly reduced the TG content in a dose-dependent manner. In db/db mice, 4 weeks of CA treatment at 20 mg/kg/day significantly decreased body weight gain and the blood glucose level of db/db mice. CA treatment also improved the serum lipid profile of db/db mice, as indicated by lower FFA and TG levels compared to those in the NAFLD group. Most importantly, the liver weight and liver index, as well as the IHTG levels, were significantly decreased, showing that CA treatment exerted effects against NAFLD *in vivo*.

As the increased IHTG is caused by increased DNL and fatty acid uptake rates (TG synthesis) and a lower fatty acid oxidation rate (TG break down), we investigated the effect of CA on the lipogenesis and fatty acid oxidation pathways. Aiming to explore the underlying mechanisms of the effects of CA on NAFLD model animals, only the NAFLD group and CA group were included in our PCR and western blotting analyses, as comparing the differently expressed factors within these two groups would be sufficient for the demonstration.

Abundant carbohydrates are converted into fatty acids and then esterified to form TGs in the liver and adipose tissues via DNL [40]. DNL in the liver is mediated by a series of coordinated lipogenic enzymes [41]. Briefly, citrate, which is generated from glucose via glycolysis and the tricarboxylic acid cycle, is transformed by ACLY into acetyl-CoA. Acetyl-CoA from the first step of DNL is carboxylated by ACC to form malonyl-CoA. Mammals have two types of ACC proteins, ACC1 in the cytoplasm and ACC2 on the mitochondrial outer membrane [42]. Malonyl-CoA is believed to inhibit CPT1A, and suppression of ACC1 and ACC2 decreases the hepatic malonyl-CoA levels, increases fatty acid oxidation, and improves NAFLD in diet-induced rat models [43, 44]. Malonyl-CoA is further converted into palmitic acid by FAS. Palmitic acid is elongated on the endoplasmic reticulum to form LCFAs, which are subsequently desaturated by SCD1 to generate unsaturated fatty acids. Palmitic acid, LCFAs, and unsaturated fatty acids are all fatty acid products of DNL, and they can be esterified to generate IHTG [40, 44, 45]. In this study, CA downregulated the mRNA expression of the lipogenesis genes ACLY, ACC, FAS, and SCD1, suggesting that CA suppresses fatty acid synthesis *in vivo*. The western blotting results showed that CA also significantly decreased the related protein expression. As an *in vitro* model of human liver steatosis, OA-induced lipid accumulation was suppressed by CA in HepG2 cells. The results showed that 100 *μ*M of CA significantly downregulated several key genes' expression levels in lipogenesis.

The genes encoding lipogenesis proteins are primarily governed by transcription factors [6]. SREBP1c binds to sterol regulatory elements, ChREBP binds to carbohydrate response elements, and LXRs bind to LXR response elements, all located in the promoter region of lipogenesis genes, and thereby upregulate their target genes [6, 46, 47]. LXR*α* is mainly expressed in the liver and other lipogenic tissues [48] and may also activate SREBP1c and ChREBP [49, 50]. Furthermore, PPAR*γ* is also considered to be an agonist of SREBP1c, as hepatic deletion of PPAR*γ* downregulated SREBP1c, SCD1, and ACC [51]. Our experiments revealed that CA decreased the expression of transcription factors of lipogenesis genes, consistent with the downregulation of their target genes. In addition, BDK and PPM1K are two kinases that coregulate ACLY activity, and hepatic BDK overexpression may lead to excessive DNL. The BDK : PPM1K ratio is believed to be a bioindicator of DNL and metabolic disorder phenotype, and the ratio can be increased by ChREBP [52]. CA downregulated BDK and upregulated PPM1K, which led to a decreased BDK : PPM1K ratio. This may also indicate its inhibitory effect on the transcription factor ChREBP, as well as reflecting CA's therapeutic effects against obesity.

TG accumulation may also be attributed to an increased exocellular fatty acid intake rate. Fatty acids are taken up by hepatocytes through several membrane proteins such as CD36, fatty acid translocase, and fatty acid-binding proteins [53]. In obese rats, CD36 mRNA expression is positively related to the IHTG level and liver steatosis severity [54]. As PPAR*γ* promotes CD36 transcription in the liver [55, 56] and PPAR*γ* was downregulated in the CA group, we investigated the expression of its transcriptional target, CD36. The results showed that CD36 mRNA was significantly downregulated as predicted, indicating that CA may also inhibit the fatty acid intake of hepatocytes.

Fatty acids are principally consumed in the liver, via fatty acid *β*-oxidation, which mainly takes place in the mitochondria [8]. LCFAs are activated by converting them to LCFA-CoA by long-chain acyl-CoA synthetases [57] and they are then transferred to mitochondria by CPT1A [58]. PGC1*α* is a coactivator of PPAR*α*, which plays an important role in fatty acid oxidation [59]. Deletion of PPAR*α* decreased hepatic fatty acid *β*-oxidation and aggravated hepatic steatosis in mice [60]. In our db/db mice, CA treatment was shown to remarkably increase the CPT1A mRNA and protein expression, as well as increasing the mRNA expression of PGC1*α* and PPAR*α*. Additionally, CA treatment downregulated ACC2 mRNA expression, which, as discussed above, generates malonyl-CoA and inhibits the activity of CPT1A (Figure 7).

In addition, CA is believed to be of relatively low toxicity [13, 15, 22], and novel formulations are being developed to boost its bioavailability [11]. Thus, CA may be an ideal alternative treatment for NAFLD. However, further experiments, especially comprehensive investigations, such as omics investigations, are still required to explore the mechanisms of the beneficial effects in more detail. It is also necessary to determine the toxic and effective dosages of CA prior to its clinical use.

## 5. Conclusion

In conclusion, this study examined CA's effect on lipid metabolism in OA-treated HepG2 cells and mice with NAFLD and investigated the underlying mechanisms. CA showed a therapeutic effect against hyperlipidemia both *in vitro* and *in vivo*. In terms of the possible mechanisms, CA downregulated the transcription factors PPAR*γ*, SREBP, LXR*α*, and ChREBP, and their target genes ACLY, ACC, FAS, and SCD1. CA also upregulated PGC1*α*, PPAR*α*, and CPT1A and downregulated CD36. Taking all the evidence together, it is presumed that CA suppresses IHTG accumulation and ameliorates NAFLD by inhibiting lipogenesis and fatty acid intake, as well as promoting hepatic fatty acid oxidation.

## Figures and Tables

**Figure 1:** (a) Chemical structure of cinnamic acid (CA). (b) CCK-8 assay results. Control group: HepG2 cells cultured with 10% FBS in DMEM. 25 *μ*M group: cells cultured with 25 *μ*M CA, 10% FBS in DMEM. 50 *μ*M group: cells cultured with 50 *μ*M CA, 10% FBS in DMEM. 100 *μ*M group: cells cultured with 100 *μ*M CA, 10% FBS in DMEM. 200 *μ*M group: cells cultured with 200 *μ*M CA, 10% FBS in DMEM. (c) Images of oil red O staining of HepG2 cells (200X magnification). (d) Triglyceride (TG) content of HepG2 cells after treatment for 24 h. (e) mRNA expression of ATP-citrate lyase (ACLY), acetyl-CoA carboxylase 1 (ACC1), fatty acid synthase (FAS), and stearoyl-CoA desaturase 1 (SCD1), carnitine palmitoyltransferase-1A (CPT1A), and ACC2 in HepG2 cells. Normal group: cells cultured with 10% FBS in DMEM. Model group: cells cultured with 0.5 mM oleic acid (OA). 25 *μ*M group: cells cultured with 0.5 mM OA and 25 *μ*M CA. 50 *μ*M group: cells cultured with 0.5 mM OA and 50 *μ*M CA. 100 *μ*M group: cells cultured with 0.5 mM OA and 100 *μ*M CA. Data are presented as mean ± SD, ^*∗*^*p* < 0.05,  ^*∗∗*^*p* < 0.01, compared to the model group; ^#^*p* < 0.05, compared to control group.

**Figure 2:** Cinnamic acid (CA) reduced body weight gain of db/db mice, liver mass, liver index, and blood glucose levels. (a) Body weight of mice compared among groups of mice. (b) Body weight gain of mice compared to initial body weight at week 0. (c) Liver mass of mice. (d) Liver index (liver mass/body weight) of mice. (e) Blood glucose levels from week 0 (tested by portable glucose monitor using blood from tail vein) and week 4 (tested by automated chemistry analyzer using blood collected from abdominal aorta). (f) Epididymal fat (from the left side of mice) mass. Normal group: wt/wt mice treated with vehicle. NAFLD group: db/db mice treated with vehicle. CA group: db/db mice treated with CA 20 mg/kg/day. Data are presented as mean ± SD. ^*∗*^*p* < 0.05, ^*∗∗*^*p* < 0.01, compared to the model group.

**Figure 3:** Serum lipid profile and intrahepatic triglyceride (IHTG) levels in mice. Serum total cholesterol (TC) levels (a), serum triglyceride (TG) levels (b), serum high-density lipoprotein (HDL) levels (c), serum low-density lipoprotein (LDL) levels (d), serum-free fatty acid (FFA) levels (e), and IHTG levels (f) in mice. Normal group: wt/wt mice treated with vehicle. NAFLD group: db/db mice treated with vehicle. CA group: db/db mice treated with CA 20 mg/kg/day. Data are presented as mean ± SD, ^*∗*^*p* < 0.05, ^*∗∗*^*p* < 0.01, compared to the NAFLD group.

**Figure 4:** Histological observation results (200× magnification). (a) Images of H&E staining of liver tissues. (b) Images of H&E staining of epididymal fat tissues. (c) Immunohistochemical (IHC) staining of hepatic sterol regulatory element-binding protein 1c (SREPB1c) in mice. (d) IHC staining of hepatic carnitine palmitoyltransferase-1A (CPT1A) in mice. (e) Mean optical density of IHC staining images. Normal group: wt/wt mice treated with vehicle. NAFLD group: db/db mice treated with vehicle. CA group: db/db mice treated with CA 20 mg/kg/day. Data are presented as mean ± SD. ^*∗*^*p* < 0.05, ^*∗∗*^*p* < 0.01, compared to the NAFLD group.

**Figure 5:** Cinnamic acid (CA) downregulated lipogenic transcription factors and other lipogenic genes in db/db mice. (a) Protein expression of ATP-citrate lyase (ACLY), acetyl-CoA carboxylase (ACC), fatty acid synthase (FAS), and stearoyl-CoA desaturase 1 (SCD1) in db/db mice assessed by western blotting. (b) mRNA expression of ACLY, ACC1, FAS, SCD1, sterol regulatory element-binding protein 1c (SREBP1c), carbohydrate-responsive element-binding protein (ChREBP), liver X receptor *α* (LXR*α*), peroxisome proliferator-activated receptor *γ* (PPAR*γ*), branched-chain ketoacid dehydrogenase kinase (BDK), and branched-chain ketoacid dehydrogenase phosphatase (PPM1K) in db/db mice assessed by qPCR. NAFLD group: db/db mice treated with vehicle. CA group: db/db mice treated with CA 20 mg/kg/day. Data are presented as mean ± SD, *n* = 3 for western blotting analyses, *n* = 5 for PCR analyses. ^*∗*^*p* < 0.05, ^*∗∗*^*p* < 0.01, compared to the NAFLD group.

**Figure 6:** CA upregulated the fatty acid oxidation pathway and reduced CD36 mRNA expression in db/db mice. (a) Protein expression of carnitine palmitoyltransferase-1A (CPT1A) in db/db mice assessed by western blotting. (b) mRNA expression of CPT1A, acetyl-CoA carboxylase 2 (ACC2), peroxisome proliferator-activated receptor *α* (PPAR*α*), peroxisome proliferator-activated receptor-*γ* coactivator 1*α* (PGC1*α*), and CD36 in db/db mice assessed by qPCR. NAFLD group: db/db mice treated with vehicle. CA group: db/db mice treated with CA 20 mg/kg/day. Data are presented as mean ± SD, *n* = 3, for western blotting analyses, *n* = 5 for PCR analyses. ^*∗*^*p* < 0.05, ^*∗∗*^*p* < 0.01, compared to the NAFLD group.

**Figure 7:** Effect of cinnamic acid (CA) on hepatic lipid metabolism pathways investigated in this study. According to this study, in hepatocytes, CA downregulates the following factors: ATP-citrate lyase (ACLY), acetyl-CoA carboxylase 1 (ACC1), ACC2, fatty acid synthase (FAS), stearoyl-CoA desaturase 1 (SCD1), sterol regulatory element-binding protein 1c (SREBP1c), carbohydrate-responsive element-binding protein (ChREBP), liver X receptor *α* (LXR*α*), peroxisome proliferator-activated receptor *γ* (PPAR*γ*), branched-chain ketoacid dehydrogenase kinase (BDK), and CD36. CA upregulates the following factors: branched-chain ketoacid dehydrogenase phosphatase (PPM1K), carnitine palmitoyltransferase-1A (CPT1A), peroxisome proliferator-activated receptor *α* (PPAR*α*), and peroxisome proliferator-activated receptor-*γ* coactivator 1*α* (PGC1*α*). The suppressed lipogenesis decreased fatty acid intake and boosted fatty acid oxidation contribute to the decreased triglyceride (TG) level in the liver. LCFA: long-chain fatty acid; FFA: free fatty acid; ↑: upregulated; ↓: downregulated.

**Table 1:** Sequences of primers used in RT-qPCR.

Gene	Forward primer	Reverse primer
ACC1	GATGAACCATCTCCGTTGGC	GACCCAATTATGAATCGGGAGTG
ACC2	CGCTCACCAACAGTAAGGTGG	GCTTGGCAGGGAGTTCCTC
ACLY	ACCCTTTCACTGGGGATCACA	GACAGGGATCAGGATTTCCTTG
BDK	ACATCAGCCACCGATACACAC	GAGGCGAACTGAGGGCTTC
CD36	ATGGGCTGTGATCGGAACTG	GTCTTCCCAATAAGCATGTCTCC
ChREBP	GAACCGCCTCTTCTGCT	CAACTCCATACAACCCTCG
CPT1A	AGATCAATCGGACCCTAGACAC	CAGCGAGTAGCGCATAGTCA
FAS	GGAGGTGGTGATAGCCGGTAT	TGGGTAATCCATAGAGCCCAG
GAPDH	AAGATGGTGAAGGTCGGTGT	GCTTCCCATTCTCAGCCTTG
LXR*α*	CTCAATGCCTGATGTTTCTCCT	TCCAACCCTATCCCTAAAGCAA
PGC1*α*	TTCAAGATCCTGTTACTACT	ACCTTGAACGTGATCTCACA
PPAR*α*	ACGCGAGTTCCTTAAGAACCTG	GTGTCATCTGGATGGTTGCTCT
PPAR*γ*	GGAAGACCACTCGCATTCCTT	GTAATCAGCAACCATTGGGTCA
PPM1K	TTATCAGCGGCCTTCATTACTTT	GGATGGAGCTTAACAACACTCTC
SCD1	TTCTTGCGATACACTCTGGTGC	CGGGATTGAATGTTCTTGTCGT
SREBP1c	CAAGAAGCGGATGTAGTCG	GAGCCGTGGTGAGAAGC
GAPDH (human)	GGAGCGAGATCCCTCCAAAAT	GGCTGTTGTCATACTTCTCATGG
ACC1 (human)	ATGTCTGGCTTGCACCTAGTA	CCCCAAAGCGAGTAACAAATTCT
ACC2 (human)	CAAGCCGATCACCAAGAGTAAA	CCCTGAGTTATCAGAGGCTGG
ACLY (human)	TCGGCCAAGGCAATTTCAGAG	CGAGCATACTTGAACCGATTCT
CPT1A (human)	TCCAGTTGGCTTATCGTGGTG	TCCAGAGTCCGATTGATTTTTGC
FAS (human)	AAGGACCTGTCTAGGTTTGATGC	TGGCTTCATAGGTGACTTCCA
SCD1 (human)	TCTAGCTCCTATACCACCACCA	TCGTCTCCAACTTATCTCCTCC

## Data Availability

The datasets used and/or analyzed during the current study are available from the corresponding author on reasonable request. A preprint of the manuscript has previously been published [61].

## Abbreviations

ACC: Acetyl-CoA carboxylase
ACLY: ATP-citrate lyase
BDK: Branched-chain ketoacid dehydrogenase kinase
BSA: Bovine serum albumin
CA: Cinnamic acid
ChREBP: Carbohydrate-responsive element-binding protein
CMC: Carboxymethyl cellulose
CPT1A: Carnitine palmitoyltransferase-1A
DAB: 3,3′-Diaminobenzidine
DNL: *De novo* lipogenesis
EDTA: Ethylenediaminetetraacetic acid
FAS: Fatty acid synthase
FFA: Free fatty acid
GAPDH: Glyceraldehyde 3-phosphate dehydrogenase
HDL: High-density lipoprotein
IHTG: Intrahepatic triglyceride
LCFA: Long-chain fatty acid
LDL: Low-density lipoprotein
LXRs: Liver X receptors
NAFLD: Nonalcoholic fatty liver disease
PGC1*α*: Peroxisome proliferator-activated receptor-*γ* coactivator 1*α*
PPAR*α*: Peroxisome proliferator-activated receptor *α*
PPAR*γ*: Peroxisome proliferator-activated receptor *γ*
PPM1K: Branched-chain ketoacid dehydrogenase phosphatase
RIPA: Radioimmunoprecipitation assay
SCD1: Stearoyl-CoA desaturase 1
SREBP1c: Sterol regulatory element-binding protein 1c
TC: Total cholesterol
TG: Triglyceride.
